# The Acceptability of Internet-Based Treatment and Characteristics of an Adult Sample with Obsessive Compulsive Disorder: An Internet Survey

**DOI:** 10.1371/journal.pone.0020548

**Published:** 2011-06-03

**Authors:** Bethany M. Wootton, Nickolai Titov, Blake F. Dear, Jay Spence, Alice Kemp

**Affiliations:** 1 School of Psychiatry, University of New South Wales, Australia; 2 Department of Psychology, Macquarie University, New South Wales, Australia; 3 Clinical Research Unit for Anxiety and Depression (CRUfAD), St Vincent's Hospital, Sydney, New South Wales, Australia; 4 Centre for Emotional Health, Department of Psychology, Macquarie University, New South Wales, Australia; University of Granada, Spain

## Abstract

**Background:**

Obsessive-compulsive disorder (OCD) is a disabling anxiety disorder, but most individuals delay seeking treatment. Internet-based cognitive behavioural therapy (iCBT) is an innovative service delivery method that may help to improve access to care, but the acceptability to consumers of such programs has not yet been established.

**Methodology:**

People with symptoms of OCD were invited to complete an online survey enquiring about demographic characteristics, symptom severity, and acceptability of Internet-based treatment. Demographic and symptom severity data were compared with people with OCD identified in a national epidemiological survey and with a sample of patients with OCD from a specialist outpatient anxiety clinic.

**Participants:**

129 volunteers to an online Internet survey, 135 patients at a specialist anxiety disorders outpatient clinic, and 297 cases identified in a national epidemiological survey.

**Main Measures:**

Demographic characteristics, and severity of symptoms as measured by the Kessler 10-Item scale, the 12-item World Health Organisation Disability Assessment Schedule - Second Edition and the Yale Brown Obsessive Compulsive Scale - Self Report Version.

**Principal Findings:**

The Internet sample was similar demographically but reported more severe symptoms than the comparison groups, although had similar severity of symptoms of OCD compared with other clinical samples reported in the literature. Participants reported Internet-based treatment for OCD would be highly acceptable.

**Conclusions:**

Internet-based treatment may reduce barriers to accessing treatment to people with OCD. Individuals in this study were similar demographically to other samples and had similar severity of symptoms as those identified in other clinical samples, suggesting that Internet-based treatment using techniques employed in face-to-face treatment may be effective in this group. Internet-based treatments for OCD need to be developed and evaluated.

## Introduction

Obsessive-compulsive disorder (OCD) is an anxiety disorder characterized by intrusive, unwanted and ego-dystonic obsessions and/or compulsions. It has a 12-month prevalence of 2% [1], is highly co-morbid with other psychiatric disorders, and results in considerable disability [2]. Obsessive-compulsive disorder can be treated successfully with cognitive behavioural treatment (CBT), particularly exposure with response prevention [3], [4], [5], [6].

Despite the disability associated with symptoms, most individuals with OCD delay seeking treatment for at least 10 years from onset of symptoms [7]. Barriers to treatment seeking in this population are similar to those relevant to other anxiety disorders, and include the direct and indirect costs of treatment, the limited number of mental health professionals skilled in the treatment of anxiety disorders, and stigma [8], [9], [10]. Stigma and shame about symptoms are particularly relevant to subgroups of people with OCD who experience obsessions characterized by sexual, religious, or aggressive themes. Unfortunately, less than half of those with OCD who seek treatment receive an evidence-based intervention [11], [12]. Interventions that can improve access to evidence-based treatments for people with OCD are urgently required.

A recent innovative approach that may improve access to evidence-based care for people with anxiety disorders is the use of Internet-based cognitive behavioral therapy (iCBT) programs. iCBT involves the administration of highly structured online lessons that present the same information and skills typically taught in face-to-face CBT, often with telephone-based or email support from a trained support person or clinician [13]. The results of recent meta-analyses of iCBT and computerised CBT indicate that these treatments produce superior effect sizes over control conditions for several anxiety disorders [14], [15], but presently there is limited evidence for the efficacy of Internet-based treatment or computerized treatments specifically for OCD [5], [16], [17], [18].

While clinical effectiveness is important, the acceptability of iCBT is an additional criterion likely to affect implementation. Acceptability refers to the degree that patients, clinicians or others are comfortable or at ease with a service and are willing to use it [19]. Clinician attitudes towards Internet or computer-based treatments are still largely neutral [20], [21], [22] or unfavorable [23]. However, the data emerging from clinical trials and online surveys indicates iCBT for anxiety and depressive disorders appears to be more acceptable to consumers [22], [24], [25] and that consumers appear willing to try Internet-based psychotherapy [22], [26]. Nevertheless, there is limited research regarding the acceptability of such interventions specifically for treating OCD.

The aims of the present study were to: 1) Examine the acceptability of Internet-based treatment for OCD to a sample of Australian adults with OCD who completed an Internet-based survey, and; 2) Compare the characteristics of respondents to the Internet survey with a sample of people with OCD who had sought face-to-face treatment at a specialist outpatient clinic and a sample of people with OCD identified in a national survey. This information will help determine whether there is demand for iCBT programs from people with OCD. Based on recent results of a similar comparison of people with anxiety and depressive disorders [27], it was expected that the Internet sample would have more severe symptoms than those identified in the national survey, but similarly severe symptoms to those attending an outpatient clinic. It was also expected that respondents to the Internet survey would rate Internet delivered treatment for OCD as an acceptable treatment option.

## Methods

### Participants

Three groups of people with symptoms of OCD were compared. Participants in all three groups were at least 18 years of age, and either met diagnostic criteria for OCD determined by a standardized diagnostic interview or were likely to meet criteria based on their scores on an OCD-specific diagnostic screening questionnaire. Across all three groups the diagnosis of OCD need not have been their principal diagnosis.

The Internet Survey group (IS) comprised respondents to an Internet survey developed for this study (see details below). This sample (n = 129) was restricted to people who were over the age of 18, were living in Australia and reported OCD symptoms that were of at least moderate severity, meeting criteria for a probable diagnosis of OCD based on a score of ≥16 on the Yale Brown Obsessive Compulsive Scale - Self Report (YBOCS-SR) [28], [29].

The second group comprised patients in an existing database from the Anxiety Disorders Clinic, St Vincent's Hospital, Sydney, Australia (ADC Group; ADC), a specialist outpatient clinic. The sample consisted of 135 individuals who received face-to-face treatment for OCD between 2005 and 2010. A diagnosis of OCD was assigned using the Computerized Composite International Diagnostic Interview 2.1 (CIDI 2.1) [30].

The third group comprised 297 individuals meeting criteria for a diagnosis of OCD identified in the 2007 Australian National Survey of Mental Health and Wellbeing. This survey was conducted by the Australian Bureau of Statistics between August and December 2007 [1] (National Survey Group; NS), included 8841 Australian residents aged 16–85 years (response rate of 60%) and derived data on lifetime mental disorders using the CIDI 3.0 [31]. We selected an unweighted subsample of respondents who met DSM-IV diagnostic criteria for lifetime OCD and who reported having symptoms in the last 12 months.

### Internet Survey Design, Development and Administration

The Internet-administered survey was developed as an “open” survey, using a convenience sampling method. Visitors to the VirtualClinic website (www.virtualclinic.org.au), a research website operated by the University of New South Wales and St Vincent's Hospital, were invited to participate. Participation was voluntary.

The questionnaire comprised 3 sections. Section 1 enquired about demographics. Section 2 included questionnaires measuring symptoms of OCD, psychological distress, and disability (see below). Section 3 enquired about the perceived advantages, perceived disadvantages, and acceptability of Internet treatment of OCD. Questions about advantages and disadvantages of Internet treatment were based on questions used in similar surveys and research [22], [24], [25]. Acceptability of Internet-based treatment was determined with the following questions, which utilized Likert-type answers: *Do you think that therapy for OCD delivered via the Internet would be effective?* (5 point scale ranging from *symptoms will get a lot worse* to *symptoms will get a lot better*), and; “If you were seeking treatment would you try treatment for OCD delivered via the Internet?” (4 point scale ranging from *definitely would* to *definitely would not*).

All participants received items in the same order and were able to change responses before submitting the survey. The questions and functionality of the survey was pilot tested on two occasions with a small non-clinical convenience sample of mental health clinicians (n = 5) and lay people (n = 5). The aim of the piloting was to examine comprehension, interpretability and functionality. Piloting was conducted in a two stage process and questions were subsequently modified after each stage. No formal analyses of internal reliability or validity were conducted.

This study was approved by the Human Research Ethics Advisory Committees of the University of New South Wales and St Vincent's Hospital, New South Wales, Australia. All participants were provided information about the study and completed a consent form before beginning the survey. No incentives were offered for participating, but respondents were invited to contact the investigator to request a copy of the final results. IP addresses of participants' computers were used to prevent users from repeating the survey. The survey took an average 15 minutes to complete and data from the IS group was collected between May and October 2010 (22 weeks).

### Internet Survey Measures

The following measures were administered online during the Internet survey:

#### Yale Brown Obsessive Compulsive Scale, Self Report; YBOCS-SR [28]

The YBOCS-SR is a 10-item questionnaire that measures the severity of OCD symptoms independently of the type of obsessions and compulsions the individual experiences. Each item is measured on a 5-point scale, with 0 indicating *no symptoms* and 4 *extreme symptoms*. The range for the total YBOCS-SR is 0–40, with higher scores indicating greater severity of OCD symptoms. The self-report scale has high internal consistency [10], [32], [33], [34] and the internal consistency in the current study was high (Cronbachs alpha = .72). Using a cut off of 16, the sensitivity of the YBOC-SR is excellent and ranges from 94–100% [29], [34]. Scores on the YBOCS-SR are only available for the Internet Group.

#### The Kessler 10 (K-10) [35]

The K-10 is a brief self-report measure of non-specific psychological distress. Scores are rated on a 5-point Likert scale and higher scores indicate higher distress. Scores are summed and range from 10 to 50. The scale has excellent internal consistency with a Cronbach's alpha of 0.92 [35]. The internal consistency in this study was excellent (Cronbachs alpha = .91). Scores on the K-10 are available for all three groups.

#### World Health Organization Disability Assessment Schedule II (WHODAS-II) [36]

The WHODAS-II is a measure of general functioning and disability. The WHODAS-II is measured on a 5-point Likert scale (1–5) and total scores range from 12 to 60 with higher scores indicating higher levels of disability. The WHODAS-II has a reported internal consistency of 0.86 and high test-retest reliability [37]. The internal consistency (Cronbach's alpha) in this study was .91. Scores on the WHODAS-II are available for all three groups.

The comparator groups were also administered the K-10 and WHODAS-II. The NS group were administered these questionnaires via a trained interviewer, whilst the ADC group were administered the questionnaires in paper and pencil format.

### Survey Response Rates and Analysis

Participant flow can be seen in Figure 1. Three hundred and five respondents logged into the survey, of these 236 began the survey. One hundred and four respondents were excluded because they did not complete the YBOCS-SR or scored less than 16 on the YBOCS-SR, and three individuals were excluded because they were less than 18 years of age. The resultant sample was 129 participants who reported at least moderate symptoms of OCD and were eligible for analysis in the IS group.

**Figure 1:** Survey Flow Chart.

### Analysis Plan

Differences between samples in categorical demographic variables were assessed using chi-square tests, while mean differences in age and the symptom severity scales were assessed using one-way ANOVAs. Post-hoc tests were conducted using chi-square tests for categorical variables and independent *t*-tests with adjustments for multiple comparisons were employed for analyses involving continuous variables. Participants with missing data were omitted from specific analyses where the missing values occurred. Analyses were performed using the Statistical Package for Social Sciences (SPSS) version 18.0 for Windows [38].

## Results

### Comparison of Demographic and Symptom Severity across Groups

Table 1 shows the demographic and severity data for each group. The mean age for respondents in the IS group was 34.3 (SD = 12.2), compared to 32.0 (SD = 9.8) for the ADC and 40.7 (SD = 15.5) for the NS groups. The p-value was adjusted for multiple comparisons and set at 0.016 to reduce the rate of Type I errors. There was a significant difference in age between groups (*F_(2,560)_* = 22.6, p<0.001), with those in the NS group being significantly older than those in the other groups, but no difference between the ADC and the IS groups. There was a significant difference between groups in gender (χ2(2, *N = 561*) = 11.3, p = 0.003), with more males in the ADC than in the IS and NS groups. A significant difference between groups was also found on educational achievement (χ2 (6, *N = 540*) = 62.8, p<0.001) with those in the ADC group more likely to have achieved a diploma or degree than either of the other groups. The IS group was also more likely to have achieved a higher level of qualification than the NS group. There was no significant difference between groups in marital status (χ2 (6, *N = 561*) = 11.5, p = 0.740) or employment rates (χ2 (2, *N = 535*) = 1.8, p = 0.404).

**Table 1:** Comparisons of demographic data and severity of symptoms for the Internet Survey, Anxiety Disorders Clinic and National Survey groups.

Category	Subcategory	IS (N)	IS *Mean (SD)/Percent*	ADC (N)	ADC *Mean (SD)/Percent*	NS (N)	NS *Mean (SD)/Percent*	Test Statistic	*p*-Value
***Mean Age (SD)***		129	34.3 (12.2)†	135	32.0 (9.8) ‡	297	40.7 (15.5)† ‡	F = 22.6∧	.000
***Age in Categories (%)***	18–24 Years	129	26.4	135	19.3	297	20.5	χ2 = 65.5	.000
	25–34 years		29.5		49.6		18.9		
	35–44 years		20.9		17.8		23.9		
	45–54 years		14.0		9.6		15.8		
	55–64 years		9.3		3.7		13.1		
	65+		0		0		7.7		
***Gender (% Male)***		129	28.7* †	135	48.9* ‡	297	38.7† ‡	χ2 = 11.3	.003
***Marital Status (%)***	Single/Never Married	129	51.2	135	54.1	297	43.8		
	Widowed		0.8		1.5		2.7		
	Divorced/Separated		14.0		7.4		17.8		
	Married/Defacto		34.1		37.0		35.7		
***Highest Educational Qualification (%)***	No Qualification	129	4.7* †	114	0	297	0†	χ2 = 62.8	.000
	High School		27.9†		19.3‡		42.4† ‡		
	Vocational/Other Certificate		20.9		13.2‡		24.9‡		
	Diploma/Degree or Above		46.5* †		67.5* ‡		32.7† ‡		
***Employment Status (% Employed)***		129	63.6	135	69.6	271	63.1	χ2 = .01	.510
***K-10***		119	31.9 (8.3)* †	135	28.8(7.4) * ‡	297	20.2(7.6) † ‡	F = 122.0∧	.000
***WHODAS-II***		118	30.4 (9.9)* †	135	26.9 (8.1) ‡	297	19.4(8.0) † ‡	F = 84.7∧	.000

*Significant difference between IG and ADC groups in follow-up t-tests;

† Significant difference between IG and NG groups in follow up independent t-tests;

‡ Significant difference between ADC and NG groups in follow up independent t-tests.

∧ Tested at corrected significance level of 0.016.

With respect to symptom severity, one-way ANOVAs revealed significant differences across the three groups on both the K-10 (*F_(2,550)_* = 122.0, p<0.001) and the WHODAS-II (*F_(2,549)_* = 84.7, p<0.001). Post-hoc analyses revealed that the K-10 scores of the IS group were significantly higher than both the ADC and NS groups, while the ADC had significantly higher K-10 scores than the NS group. Post-hoc analyses revealed that the IS group had significantly higher scores on WHODAS-II than the ADC and NS groups, while the ADC had significantly higher scores than the NS group. On the YBOCS-SR, which was administered only to the IS group, 78/128 (61%) of participants scored in the *moderate range* of symptoms, 46/128 (36%) in the *severe range*, and 4/128 (3%) in the *extremely severe range*.

### Internet Group: Acceptability of Internet Based Treatments for OCD

Respondents were asked to select which options from a list of potential advantages and disadvantages were important in their potential use or rejection of Internet therapy (Tables 2 and 3). The most commonly reported advantages for using Internet-based treatment were those related to *convenience*. Of the 116 respondents, 78 (67%) reported *time saving* and 73 (63%) reported *no need to travel to appointments* as the main advantages to Internet-based treatment. Other primary reasons included *reduced costs* 70/116 (60%) and *increased privacy* 65/116 (56%). Disadvantages of using Internet-based treatments were rarely endorsed. Of the 116 respondents, 11 (10%) reported *preferring face-to-face treatment*, 10 (9%) reported they perceived their problems to be *too severe for Internet based-treatment*, and 9 (8%) reported *concerns about the lack of face-to-face contact*, *not being able to communicate ideas online*, and Internet treatment *not seeming real*.

**Table 2:** Perceived advantages of Internet-based treatments reported by the Internet Survey group (N = 116).

Advantages of accessing Internet-based treatments	n	%
Reduced time	78	67.2
No need to travel to appointment	73	62.9
Reduced costs involved	70	60.3
Privacy and anonymity	65	56.0
Embarrassment related to face-to-face	38	32.8
Face-to-face therapy is too confronting	24	20.9
Face-to-face therapy did not work previously	16	13.8
I did not think my symptoms were severe enough for face-to-face	16	13.8
Face-to-face treatment not available to me where I live	15	11.3

**Table 3:** Perceived disadvantages of accessing Internet-based treatments reported by the Internet Survey group (N = 116).

Disadvantages of accessing Internet-based treatments	n	%
Prefer face-to-face	11	9.5
My problems are too complex or severe to be treated online	10	8.6
I need to be able to see the person I am talking too	9	7.8
I won't be able to communicate my ideas online	9	7.8
Internet therapy doesn't seem real	9	7.8
I don't understand what Internet therapy is	7	6.0
Don't think it will help	5	4.3
I prefer to deal with symptoms on my own	4	3.4
Embarrassed to talk about problems over the phone/email	4	3.4
Lack of time	3	2.6
Sounds too risky	3	2.6
I would prefer medication	2	1.7
My problems are not severe enough	2	1.7
Too confronting	2	1.7
Someone told me not too	0	0
Don't have adequate access to a computer/Internet	0	0

In response to the question: *Do you think therapy via the Internet would be effective?* 25/116 (22%) indicated that believed their symptoms *would get a lot better*; 68/116 (59%) indicated that *their symptoms would get a little bit better*; 19/116 (16%) indicated that *there would be no change in their symptoms*; 2/116 (2%) reported that *their symptoms would get a little worse*; and 2/116 (2%) reported they thought *their symptoms would get a lot worse*. When asked if they would be willing to try Internet therapy (*If you were seeking treatment would you try treatment for OCD delivered via the Internet?*) 61/116 (53%) of the IS participants indicated that they *definitely would*, 38/116 (33%) indicated they *possibly would*, 15/116 (13%) indicated that they *maybe would* and 2/116 (2%) indicated that they *definitely would not* use Internet therapy.

## Discussion

The aims of the present study were to examine the acceptability of Internet-based treatment to a sample of Australian adults with OCD and to compare the characteristics of that sample with two other groups of people with OCD. All participants met diagnostic criteria for OCD during structured diagnostic assessments or were likely to meet criteria based on a psychometrically established cut-off on a measure of OCD symptom severity.

### Comparison of Demographic Characteristics and Symptom Severity

Respondents to the Internet survey with OCD were similar in their marital status and employment levels as the national and outpatient samples. The outpatient sample had the highest level of education, followed by the Internet sample and then the national sample. A similar pattern was found for age; the outpatient sample was youngest, followed by the Internet sample, and then the national sample. The only demographic characteristic on which the Internet sample differed from the other groups was gender, with the Internet sample being comprised of more females. We conclude that the Internet sample are generally representative of the wider population of those with OCD, albeit slightly younger and with a slightly greater proportion of females.

Consistent with the results of a previous comparison of an Internet sample with an outpatient and a national sample [27], the Internet sample and outpatient sample in the present study had significantly greater levels of psychological distress and disability than people in the national sample. Moreover, the severity of OCD symptoms in the Internet sample, as measured the YBOCS-SR (M = 22.71; SD = 4.7), was similar to those reported in face-to-face clinical samples (M = 22.50–26.00) [32], [39], [40]. For example, the YBOCS scores observed in this sample were similar to those reported for patients starting the BT STEPS program [17]. These results indicate that the Internet sample had non-trivial symptoms and are comparable to those who seek face-to-face treatment.

### Acceptability of Internet Treatment for OCD

Overall, respondents to the Internet survey endorsed Internet treatment for OCD as an acceptable form of treatment. This is consistent with other recent studies indicating consumers are prepared to try Internet treatment for anxiety and depression [22], [26] although to our knowledge, this is the first study to enquire specifically from people with OCD.

Ninety-eight percent of respondents indicated that they would *definitely, possibly* or *maybe* try Internet-based treatment for OCD. More than 50% of respondents endorsed reasons associated with convenience, reduced costs, and privacy and anonymity as potential advantages of using Internet-based treatment. Potential disadvantages of Internet-based treatment included preferring face-to-face treatment, perceiving one's problems as being too severe and concerns about the lack of non-verbal communication. However, these disadvantages were reported by less than 10% of the sample.

### Limitations

The main limitation of this study was the use of a convenience sample of Internet users who were visiting a clinical research website. It is likely this sample had a pre-existing favourable impression of Internet treatments, and would be expected to find such an approach acceptable. However, the demographic similarities between the Internet and national samples provides some indication that Internet treatment programs for OCD may be attractive to a more general sample. Secondly, while used for pragmatic reasons, the use of different methods for determining probable OCD diagnoses or caseness across the samples used represents a potential limitation. Nevertheless the CIDI-auto, CIDI and the use of a cut-score (i.e. >16) on the YBOC-SR are widely recognised as reliable indicators of caseness and frequently used within the literature [29], [34]. Thirdly, it is possible that respondents were not fully aware of what Internet therapy involved when answering questions about the acceptability of such treatments for OCD, and lastly, the methods of recruitment and delivery of questionnaires differed across the groups, which may introduce a level of bias to the results.

### Conclusions

Australian respondents to an Internet survey were demographically similar to those identified in a national survey and had symptoms as severe as those identified in other clinical samples. This suggests that Internet-based treatment using techniques used in face-to-face treatment may be effective in an Internet sample. Respondents to the survey reported they were willing to try Internet-based treatment. These data are of interest to policy makers, funding bodies, and developers of iCBT programs. While there are iCBT programs for other anxiety disorders there is a dearth of such programs for OCD. To date BT-STEPS [5], [16]–[17] is the only program that has aimed at treating OCD via a computer and, although producing promising results, more research is needed concerning online programs for OCD with the potential of increasing patient access. The results of this survey provide preliminary evidence for demand and acceptability of iCBT programs for OCD.
